# Whole thorax irradiation of non-human primates induces persistent nuclear damage and gene expression changes in peripheral blood cells

**DOI:** 10.1371/journal.pone.0191402

**Published:** 2018-01-19

**Authors:** Shanaz A. Ghandhi, Helen C. Turner, Igor Shuryak, Gregory O. Dugan, J. Daniel Bourland, John D. Olson, Janet A. Tooze, Shad R. Morton, Ines Batinic-Haberle, J. Mark Cline, Sally A. Amundson

**Affiliations:** 1 Center for Radiological Research, Columbia University Medical Center, New York, New York, United States of America; 2 Wake Forest Baptist Medical Center, Medical Center Boulevard, Winston-Salem, North Carolina, United States of America; 3 Department of Radiation Oncology, Duke University Medical Center, Durham, North Carolina, United States of America; ENEA Centro Ricerche Casaccia, ITALY

## Abstract

We investigated the cytogenetic and gene expression responses of peripheral blood cells of non-human primates (NHP, *Macaca mulatta*) that were whole-thorax irradiated with a single dose of 10 Gy. In this model, partial irradiation of NHPs in the thoracic region (Whole Thorax Lung Irradiation, WTLI) allows the study of late radiation-induced lung injury, while avoiding acute radiation syndromes related to hematopoietic and gastrointestinal injury. A transient drop in circulating lymphocytes and platelets was seen by 9 days, followed by elevations in respiratory rate, circulating neutrophils, lymphocytes, and monocytes at 60–100 days, corresponding to computed tomography (CT) and histologic evidence of pneumonitis, and elective euthanasia of four animals. To evaluate long-term DNA damage in NHP peripheral blood lymphocytes after 10 Gy WTLI, we used the cytokinesis-block micronucleus (CBMN) assay to measure chromosomal aberrations as post-mitotic micronuclei in blood samples collected up to 8 months after irradiation. Regression analysis showed significant induction of micronuclei in NHP blood cells that persisted with a gradual decline over the 8-month study period, suggesting long-term DNA damage in blood lymphocytes after WTLI.

We also report transcriptomic changes in blood up to 30 days after WTLI. We isolated total RNA from peripheral blood at 3 days before and then at 2, 5 and 30 days after irradiation. We identified 1187 transcripts that were significantly changed across the 30-day time course. From changes in gene expression, we identified biological processes related to immune responses, which persisted across the 30-day study. Response to oxygen-containing compounds and bacteria were implicated by gene-expression changes at the earliest day 2 and latest, day 30 time-points. Gene expression changes suggest a persistent altered state of the immune system, specifically response to infection, for at least a month after WTLI.

## Introduction

The Non-Human Primate (NHP) is the most appropriate model for the study of radiation response and injury, as well as for assessing the effect of mitigators of acute radiation syndrome (ARS) and lung Delayed Effects of Acute Radiation Exposure (DEARE) [1]. The NHP model has advantages over small animal models, as it more closely resembles human physiology, size and longevity; and studies of health effects of radiation exposure in NHPs address the need for transferability of large-animal study results to humans [2]. NHPs mimic humans in many ways including similarities in genome, neuroanatomy, neurophysiology, immunogenetics, and age-related changes in immune function [3, 4]. NHPs also share similar hematopoietic stem cell dynamics, engraftment properties, and cytokine requirements with humans [5, 6]. Studies of the genome of *Macaca mulatta* have revealed 93% sequence similarity between *M*. *mulatta* and *H*. *sapiens*. Positive selection of genes in the human genome appear to be enriched in biological functions related to immune response and signal transduction [7], making *M*. *mulatta* a relevant NHP model for molecular studies and cytogenetic analyses [8].

Total body irradiation (TBI) studies in mice and NHPs have provided critical information related to the changes associated with ARS, specifically tissue damage and organ failure in addition to diagnostic endpoints such as blood cell counts and respiratory rates. In a highly comprehensive and systematic review, MacVittie *et al* [9] provide a detailed comparison of fifteen independent studies of TBI of NHPs with and without medical management including mitigation of hematopoietic effects. These studies have begun to establish dose-response relationships for induction of Hematopoietic ARS (H-ARS, 7.2–8.9 Gy) [10] and Gastro-Intestinal ARS (GI-ARS, 10–14 Gy) [11] in NHP by total body irradiation. In another study, NHP were exposed to TBI doses between 6.25 and 8.75 Gy to investigate H-ARS within the first 60 days following TBI; neutropenia, lymphopenia and loss of platelets were observed to occur within 2 weeks after irradiation [12].

With the use of *in vivo* TBI studies in NHP and mouse models, a number of candidate countermeasures have been developed to mitigate both hematopoietic and GI injury in acute radiation syndrome (summarized in [13]). With the help of such mitigators, especially in a more realistic nuclear or radiological event scenario where partial shielding may occur and dose is non-uniform, there is an increased probability of surviving H-ARS and GI-ARS. This in turn increases the probability of late development of multi-organ failure radiation sub-syndromes such as cutaneous and lung injury [13, 14].

The lung is a particularly radiosensitive organ in humans. From radiation studies in patients with metastatic cancer receiving upper partial-body irradiation, development of lung injury in the form of pneumonitis occurred after an 8 Gy dose of radiation [14, 15]. The Medical Countermeasures against Radiological Threats (MCART) Consortium therefore established an animal model platform in compliance with the FDA Animal Rule for testing medical countermeasures for the treatment of ARS and prolonged effects of radiation including lung DEARE [1, 16]. Both mouse and NHP models were established that comprise a more realistic model of radiation response and its sequelae compared to Total Body Irradiation (TBI), and these are called Partial Body Irradiated with Bone Marrow sparing (PBI/BM) models. A study in the PBI/BM5 (Partial Body Irradiation with 5% bone marrow sparing) NHP model performed by MacVittie *et al*. [17] has extensively characterized the radiation-induced lung and gastro-intestinal damage in addition to changes in blood sub-populations. All doses of PBI/BM5 caused neutropenia and thrombocytopenia with full recovery by 30 days and 60 days post irradiation, respectively.

To address radiation-induced lung injury and mitigation, the Whole Thorax Lung Irradiation (WTLI) model was established, in which a dose of radiation is targeted at the mid-point of the thorax, irradiating both lung and heart [14, 18]. Our study focused on WTLI of NHP and long-term changes in peripheral blood at the cytogenetic and transcriptomic levels; and was part of a larger study of a novel mitigator of lung injury. The mitigator study investigates the role of a manganese porphyrin based mimic of superoxide dismutase, Mn (II) *meso*-tetrakis (*N*-n-hexylpyridinium-2-yl) porphyrin, MnTnHex-2-PyP^5+^ [19]. Its analog, MnTnBuOE-2-PyP^5+^ (BMX-001) is in two clinical trials on the radioprotection of normal tissue in glioma and head & neck cancer patients (NCT02655601 and NCT02990468). In our arm of the study, NHPs were exposed to a high-dose partial body exposure of 10 Gy x-rays, which is an LD_70/180_ (a lethal dose to 70% of the population in 180 days) in the NHP-WTLI model [14, 18]. All animals developed pneumonitis after WTLI irradiation at this dose.

The cytokinesis-blocked micronucleus assay (CBMN) is one of the most commonly used and best-validated methods for measuring chromosome damage in peripheral blood lymphocytes [20, 21] and also one of the few available techniques with the required characteristics of sensitivity, specificity, transportability, and reproducibility to be an effective biological dosimeter of ionizing radiation exposure [22]. The measurement of DNA damage in cultured human and/or mammalian cells is specifically restricted to once-divided binucleate (BN) cells, which are the cells that express MNi [21]. Micronuclei (MNi) result from acentric chromosome fragments or whole chromosomes lagging behind during anaphase. Radiation-induced micronuclei in peripheral blood lymphocytes (PBLs) strongly correlate with dose and radiation quality. With a half-life of about a year, micronucleus formation is a proven long-term biomarker for the evaluation of *in vivo* radiation exposure of occupationally, medically and accidentally exposed individuals [23].

Gene expression studies following radiation in human blood [24–26], mice [27–29] and NHPs [30–32]; are a well-established approach for understanding the mechanism and regulation of the radiation response. In addition, transcriptomic studies have been useful in identifying candidate targets for radiation biodosimetry, using biofluids such as blood and serum across species [24, 33, 34] and using different modes and types of radiation. We were interested in the long-term cytogenetic and gene expression response of blood cells to radiation in a large animal model after partial body irradiation. Therefore, we investigated changes in micronucleus frequency and transcriptomic changes after 10 Gy to the NHP whole thorax. Measurement of MNi yields in the blood lymphocytes after initial radiation exposure showed a significant induction of MNi that persisted with a gradual decline over the 8-month study period. Gene expression changes at 2, 5 and 30 days post-radiation showed that although individual genes responded differently over the 30-day time course, biological processes and function enrichment analysis suggested a persistent alteration of the immune system, specifically in processes related to fighting infection. This is the first study to report the cytogenetic damage and transcriptomic changes in blood cells following partial body irradiation in NHP using the Whole Thorax Lung Irradiation (WTLI) model, and the results will be helpful to understand the effect of radiation on the physiological changes in blood cells during the progression of lung DEARE.

## Materials and methods

### Animals and irradiation

Nine male Rhesus macaques (*Macaca mulatta*) of Chinese genetic origin, aged 3.75 to 9.25 years (mean age = 5.59 years) and ranging from 4.2 to 10.3 kg in weight (mean weight = 6.51 kg) were sourced from Primate Products (Immokalee, FL) for this study. All procedures in this study were performed at Wake Forest University, in accordance with the recommendations in the Animal Welfare Act and the Guide for the Care and Use of Laboratory Animals of the National Institutes of Health [35]. The protocol was approved by the Association for Assessment and Accreditation of Laboratory Animal Care and approved by the Wake Forest University Institutional Animal Care and Use Committee (Animal Welfare Assurance Number A-3391-01). All efforts were made to minimize suffering. Animals were housed with visual and limited physical contact with other monkeys, and were fed a diet mimicking the North American Diet (5LOP, LabDiet, St. Louis, MO) with the addition of fruit and vegetables and a variety of environmental enrichments on a daily basis. These animals were part of a larger study on the mitigation of radiation-induced lung injury. We obtained samples at pre- and post-irradiation times for our study on radiation induced gene expression and cytogenetic changes in blood. Animals reaching pre-determined humane endpoints (respiratory rate > 100 breaths per min) were humanely euthanized by sedation (ketamine, 15 mg/kg) followed by anesthesia to a deep surgical plane by intravenous pentobarbital (to effect, typically > 30 mg/kg), followed by exsanguination. Complete necropsy examinations with histopathologic examinations were done for all animals.

A clinical linear accelerator, calibrated according to national standards for human radiation treatment, was used for all irradiations. A 6 MV x-ray, two-field, parallel-opposed, isocentric technique was used with anterior (AP) and posterior (PA) fields. Each oblong field (13.0 cm long (4.0 cm, 9.0 cm) x 12.0 cm wide) covered the lungs from the superior aspect to 4 cm inferior to the xyphoid and laterally with 2 cm of flash beyond the right and left skin surfaces. Average AP-PA diameters for 3 groups (sizes) of animals were used to calculate the amount of beam time in monitor units (MU), and a physical wedge was used in the AP field (heel superior; angle of 10 to 30 degrees, determined for each animal) as a missing tissue compensator for improved dose homogeneity at the mid-plane. Dose calculations were performed for homogenous (water-equivalent) tissue based on the AP-PA diameters, without tissue heterogeneity considerations. The fields were equally weighted to deliver 5 Gy each to the AP-PA midline for a total of 10 Gy, with a nominal dose rate typically used for human radiation treatment of 6 Gy/min (600 MU/min) at the isocenter.

Each NHP was anesthetized with ketamine (5–15 mg/kg, subcutaneously) and dexmedetomidine (0.0075–0.015 mg/kg, subcutaneously) and was breathing ambient air. The anesthetized animal was placed in the irradiation position on the flat linear accelerator table, arms up over the head, lightly restrained, with the central axis of the anterior field at the level of the xyphoid. The AP field was then imaged to confirm position (6 MV x-ray beam with electronic portal imaging device (EPID)) followed by the same imaging to confirm position for the opposed, PA field. The PA field was then irradiated (5 Gy) and the linear accelerator rotated back 180 degrees for irradiation of the AP field (5 Gy). The irradiation procedure, including animal positioning, portal imaging and irradiation took approximately 18 minutes per animal, with an irradiation time of approximately 3 minutes (PA: 1 min; AP: 2 min).

Respiratory rates were measured daily by cage-side observation of awake animals. Animals were assessed at least twice daily for evidence of respiratory distress. Whenever animals were sedated, continuous monitoring of heart and respiratory rates and SpO2 by pulse oximetry were done. Data were collected from non-sedated animals observed in their home enclosure. Animals were euthanized when the respiratory rate increased to more than 100 breaths per minute. Antibiotics and steroids were not administered as part of treatment for these animals. Animals received supportive care, subcutaneous fluids and non-inflammatories (ketoprofen 3–5 mg/kg buprenorphine 0.01 mg/kg IM) as needed based on pain scores and clinical pathology.

### Blood collection and counts

Peripheral blood samples (~ 1 mL) were collected in lithium-heparin vacutainer tubes (Becton-Dickson, Franklin Lakes, New Jersey) and PAXgene RNA stabilization tubes (PreAnalytix, Qiagen, catalog number 762165). For the micronucleus assay, blood was collected over the 8-month study period (Days -3, 2, 5, 37, 66, 93, 123, 151, 186 and 249). Fresh blood samples were shipped FedEx priority overnight at ambient temperature to the Center for Radiological Research, Columbia University Medical Center, New York, NY. During the winter months, a heat pack was included with the blood shipment. Blood differentials were measured from separate EDTA tubes (Becton-Dickinson) collected pre-irradiation (at 191 and 72 days before irradiation), and again at 9 days post-irradiation, and then approximately weekly from this time point until 4 months post-irradiation, at which time blood counts were measured once a month until 8 months. Total and differential blood counts were done by a veterinary reference laboratory (IDEXX, North Grafton, MA). Analyses of blood cell counts were performed by using the Dunnett’s method to adjust for comparison of all times to the baseline.

### Micronucleus assay

Whole blood samples (~ 1 mL) were diluted with 5 mL of RPMI-1640 medium (Invitrogen, Eugene, OR). The diluted blood mixtures were layered over an equal volume of lymphocyte separation media (Histopaque-1083; Invitrogen); then centrifuged at 1300 rpm for 30 minutes. The lymphocytes formed at the interface between the separation medium were collected using a glass pipette and then washed with 1 X phosphate buffered saline (PBS). The cells were transferred to 12-well multi-well tissue culture plates (Becton, Dickinson and Company, Franklin Lakes, NJ) containing 5 mL pre-warmed RPMI-1640 medium supplemented with 15% heat-inactivated fetal calf serum (Invitrogen), 2% Pen/Strep (10,000 units/mL penicillin and 10,000 μg/mL streptomycin; Invitrogen) and 2% phytohaemagglutinin (PHA; Invitrogen).

Cells were cultured at 37°C in a humidified atmosphere with 5% CO_2_. After 44 hours of incubation, cytochalasin B (Cyt-B, catalog number C6762, Sigma; stock solution 3000 μg/mL dissolved in dimethylsulphoxide; Sigma, St. Louis, MO) was added to the culture medium at a final concentration of 6 μg/mL. Cells were cultured for an additional 26 hours to arrest cytokinesis and induce the formation of once-divided bi-nucleated cells. To harvest lymphocytes, samples were transferred to a 15 mL tube and centrifuged at 1,000 rpm for 10 minutes and the supernatant discarded. The pelleted cells in the tube were treated for 10 minutes with cold hypotonic solution (0.075 M KCl, Sigma-Aldrich, St. Louis, MO) and fixed twice with ice-cold fixative (methanol: glacial acetic acid:: 3:1) and then stored at 4°C in a fireproof refrigerator. Prior to slide preparation, the lymphocytes were centrifuged, supernatant discarded and resuspended in ~0.5 mL of fresh fixative. A small drop of lymphocyte suspension was transferred to a clean glass slide; then allowed to air dry for 10 minutes. The nuclei were counter-stained with DAPI Vectashield^®^ mounting medium (catalog number H-1200; Vector Laboratories, Inc., Burlingame, CA). The pre-irradiation blood sample from animal NHP 001 was not collected for the CBMN assay.

### Scoring and analysis of MNi

The scoring of micronuclei per bi-nucleate (MNi/BN) cell yields was based on the Fenech scoring criteria [36]. MNi/BN yields were evaluated using a fluorescent microscope (Zeiss Axioplan 2; Carl Zeiss MicroImaging Inc., Thornwood, NY) with a 40x air objective. At least 500–1000 bi-nucleated cells were scored per sample, unless indicated otherwise.

### Statistics

Blood count data were compared over time using a mixed model ANOVA model with a fixed effect for days since irradiation and a random subject effect. As well estimating a main effect for time, all post-irradiation time points were compared to the baseline value; p-values were adjusted for multiple comparisons using Dunnett’s method. A two-sided alpha level of 0.05 was used to indicate statistical significance. All analyses of blood count data were performed in SAS (v. 9.4, Cary, NC).

For micronuclei data analyses, uncertainties (95% confidence intervals, CIs) for the fractions of bi-nucleated cells with ≥1 micronuclei observed for each NHP donor at each time after irradiation were calculated using the score confidence interval approach for Binomial proportions [37]. Logistic regression was used to model the dependence of the fraction of cells with micronuclei on time, radiation, and NHP donor. The regression was performed using R software (version 3.2.3). A two-sided alpha level of 0.05 was used to indicate statistical significance. We considered the following four model structures, arranged in order of increasing complexity: (1) pooling the data from all NHP donors and therefore allowing the fraction of cells with micronuclei to depend only on time and radiation. (2) Allowing the baseline pre-irradiation fractions of cells with micronuclei (determined by regression intercepts) to vary by NHP donor, while keeping the effects of time and radiation in common for all animals. (3) Allowing the baseline levels and the effects of time and radiation to vary by NHP. (4) Adding quadratic and interaction terms for time and radiation. Data support for these different model versions were compared using the Akaike information criterion (AIC).

### Microarrays, gene ontology and network analysis

Pre-irradiation (3 days before irradiation) and post-irradiation (at 2, 5 and 30 days) whole blood samples were drawn into PAXgene RNA stabilization solution from 8 NHP exposed to 10 Gy X-rays to the thoracic region in the no-mitigator arm of the larger study. We isolated RNA from the blood using the PAXgene Blood RNA method (catalog number 762165, PreAnalytix GmBH), and then depleted globin transcripts using the Ambion GLOBINclear-Human kit (catalog number AM1980,Life Technologies, Grand Island, NY). We evaluated the samples for RNA integrity using the Agilent 2100 Bioanalyzer and samples with RIN values > 8.0 were used for further analysis.

We processed five samples from each of the following groups: pre-irradiation, day 2, day 5 and day 30 and used the RNA for microarray hybridization. We chose five biological replicates for gene expression analyses and all changes after irradiation were compared with matched controls; with only one exception where materials were not of the required quantity and total RNA from two different animals were pooled. We used Agilent Whole Human Genome 4X44K v2 microarrays for measurement of levels of transcripts, following the Agilent recommended protocol. Previous studies have shown the usefulness of human microarray platforms for the detection of NHP gene expression [30, 38, 39]. We then used the class comparison tool in BRB Array Tools [40] using a p-value cut-off of 0.005 and False Discovery Rate (FDR) <10% to identify differentially expressed genes between groups. The data are deposited in the Gene Expression Omnibus database as GSE84898.

We further analyzed the differentially expressed genes at each time in this study using the PANTHER ver 10.0 (Protein ANalysis THrough Evolutionary Relationships) gene ontology tool [41]. Benjamini corrected p-values <0.05 were considered significant. Genes that were significantly differentially expressed from each time point were also imported into Ingenuity Pathway Analysis (IPA from Ingenuity^®^ Systems, http://www.ingenuity.com) software. In this analysis software, we used the core gene-expression analysis tool to predict networks and associations between genes and regulatory molecules based on curated information from published data. We focused our analysis on RNA, proteins and genes as potential upstream regulators with predicted involvement in the gene expression networks. IPA calculates a z score for each upstream regulator based on the number of target genes in the gene list and the type of relationship (transcriptional activation or inhibition) between the regulatory molecule and the downstream transcripts [42]. The z score is a significance measure that a regulator may be involved in gene regulation based on published literature and also indicates the activation state of a regulator. We compiled a list of transcriptional regulators with z scores of absolute value ≥ 2 for at least one time point in the time course, indicating significant activation/inhibition for at least one time point. For the 82 regulators that passed this criteria, we also included intermediate z scores (-2 > z score < 2) at other time points for analysis. An intermediate z score (-2 > z score < 2) suggests that there were gene targets within the data set downstream of the transcriptional regulator, and that the prediction was directional, but a proportion of the regulator-target relationships were inconsistent with findings in the literature. A transcriptional regulator that was not involved in upstream regulation was not assigned a z score.

### qRT-PCR measurement of mRNA levels and analysis

We prepared complimentary DNA (cDNA) from total mRNA using the High-Capacity cDNA Archive Kit (Life Technologies, Foster City, CA). Quantitative real-time RT-PCR (qRT-PCR) was performed for selected genes using Taqman^®^ assays (Life Technologies) to confirm microarray experiment findings for the selected genes. Assays used were: *IL1R1* (assay ID: Rh00991008_m1), *LY96* (assay ID: Rh01026731_m1, *MARCKSL1* (assay ID: Hs00702769_s1) and *FAIM3* (assay ID: Rh02857660_m1). 30 ng of cDNA was used as input in duplicate reactions. Quantitative real time PCR reactions were performed with the ABI 7900 Real Time PCR System using Universal PCR Master Mix (Thermofisher), with initial activation at 50°C for 120 seconds and 95°C for 10 minutes, followed by 40 cycles of 95°C for 15 seconds and 60°C for 60 seconds. Relative fold-induction was calculated by the -ΔΔCT method [43], using SDS version 2.4 (Thermofisher). Data were normalized to *GAPDH* (assay ID: Rh02621745_g1) gene expression levels, which were found to be stably expressed across all samples.

## Results

### Blood counts

Initially, lymphocyte and platelet counts declined significantly, approximately 30% from baseline by day 9 post-irradiation (p-values < 0.05), see Fig 1B and 1C. These measurements returned to base line within 24 days, by which time the mean neutrophil count had doubled (Fig 1D), rising to a 3-fold mean increase by day 66, (p-value < 0.05 for both), and corresponding to the expected pattern of radiation-induced pneumonitis. A third significant peak of neutrophilia occurred at 185 days post-exposure, disappearing by the study’s end at day 250. Animals that were euthanized later for elevated respiratory rates had higher neutrophil counts during the first 50 days of the study.

**Fig 1:** Differential blood cell counts. Total leukocyte counts (A) were most elevated at 66 days, reflecting neutrophilia (D). Transient reductions of lymphocyte counts (B) and platelets (C) were seen at day 9. Day 0 values are the overall average and SEM of the day -72 baseline measurements. * = significantly different from baseline at p<0.05 using Dunnett’s method. Error bars are 1 standard error of the mean.

### Micronucleus assay

Frequencies of micronuclei (MNi) were evaluated using the *in vitro* cytokinesis-block micronucleus (CBMN) assay and micronucleus yields per bi-nucleate cell (MNi/BN) were scored. Table 1 shows MNi frequency as the fraction of BN cells with one or more micronuclei for each NHP animal at specific time points up to 8 months after irradiation to the whole thorax. Blood samples where it was difficult to score more than 500 binucleate cells (*) and blood cultures (**) that showed no apparent mitogen-induced cell division are indicated. Four NHPs were sacrificed before the end of the study, NHP 002 (day 69), NHP 007 (day 57), NHP 008 (day 57) and NHP 009 (day 94); the trigger for euthanasia was an increase in respiratory rate to more than 100 breaths per minute. Overall, qualitative observations of the DAPI-labeled cells indicated an increased number of apoptotic and non-divided cells after radiation exposure.

**Table 1:** Micronucleus frequency in NHP peripheral blood lymphocytes measured up to 249 days post exposure.

	MNi frequency									
Day	-72	2	5	37	66	93	123	151	186	249
**NHP 001**	--	0.066*	0.060	0.049	0.065	0.055	0.067	0.058	0.056	0.067
**NHP 002**	0.033	0.049*	0.053	0.050	**	SAC				
**NHP 003**	0.038	0.062	0.063	0.062	0.061	0.066	0.052	0.067	0.061	0.058
**NHP 004**	0.041	0.058*	0.091	0.080	0.048	0.049	0.060	0.057	0.053	0.058
**NHP 005**	0.063	0.084*	0.063	0.086*	0.086	0.055	0.072	0.064	0.067	0.060
**NHP 006**	0.053	0.090	0.087	0.084	0.066	0.080	0.060	0.071	0.054	0.048
**NHP 007**	0.055	0.059*	0.067*	0.062	SAC					
**NHP 008**	0.039	**	0.071*	0.061	SAC					
**NHP 009**	0.024	0.073*	0.060*	0.076*	0.056*	0.045*	SAC			

*indicates that fewer than 500 bi-nucleated cells were scored

** indicates limited cell growth in the cell cultures

SAC denotes NHP sacrifice time.

Best-supported regression results based on AIC (Fig 2, Table 2) showed a strongly statistically significant increase in the fraction of cells with micronuclei after irradiation, which declined over time; and evidence for variation in baseline micronucleus frequencies between the NHPs. This model produced a reasonable fit to the data. Inclusion of possible donor-dependent variations in the effects of time and/or radiation, quadratic terms for time and/or radiation, or interaction terms between them, were not statistically supported based on the AIC. The results also highlight that for the surviving animals, NHP 004, NHP 005 and NHP 006; the MNi frequency remained above baseline.

**Fig 2:** Micronucleus frequency of individual animals. Logistic regression analysis of the fractions of binucleated cells with micronuclei at various times after irradiation across different NHPs. Error bars are 95% confidence intervals.

**Table 2:** Best-fit logistic regression parameter estimates for the fraction of cells with micronuclei.

Variable	Parameter estimate	Standard error	p-value
**Time (days)**	-0.0011	0.0003	2.21×10^−4^
**Radiation (Indicator)**	0.4579	0.0715	1.48×10^−10^
**NHP 001 (Intercept)**	-3.1036	0.0896	2.00×10^−16^
**NHP 002**	-0.2598	0.1151	0.0239
**NHP 003**	0.0202	0.0747	0.7867
**NHP 004**	0.0499	0.0795	0.5305
**NHP 005**	0.1841	0.0771	0.0170
**NHP 006**	0.1978	0.0740	0.0075
**NHP 007**	0.0520	0.1123	0.6432
**NHP 008**	-0.0032	0.1125	0.9773
**NHP 009**	-0.1344	0.1129	0.2339

Fig 3 shows the results from a pooled analysis for all the animals over the duration of the study. These data show similar effects of radiation and time to Fig 2. Further, the results show that the fraction of binucleated cells with micronuclei significantly increased (p-value < 0.05) after the acute 10 Gy dose followed by a slow decline up to 8 months after WTLI. As expected, the fit quality of the pooled analysis was somewhat worse than the individual analyses because the variations in baseline MNi frequencies were not accounted for. Pooled analysis, assuming no variability in the baseline MNi frequencies between animals, showed that there was a statistically significant elevation in MNi frequency even at day 249 (compared to day 0; p-value = 5.2 X 10^−3^, Pearson’s Chi-square with Yate’s correction)

**Fig 3:** Micronucleus frequency of animals (pooled samples). Mean micronucleus frequency from lymphocytes of nine irradiated NHPs, up to 8 months after WTLI. The error bars are 95% confidence intervals.

### Microarray results and gene ontology analysis

Analysis using the Agilent Whole Human Genome microarray platform showed that 1187 genes were affected in blood cells over the course of the study. Class comparisons were paired by animal, and 545, 273 and 603 genes were found to be significantly differentially expressed (p-value < 0.005 and FDR < 10%) at the mRNA level on 2, 5 and 30 days, respectively (S1 Table). A trend of increasing proportion of down-regulated genes was observed, with 20%, 32% and 57% of the differentially expressed genes down regulated at 2, 5 and 30 days, respectively. Overlap between the responding genes at various time points is shown in Fig 4 as a Venn diagram (also see S1 Table).

**Fig 4:** Venn diagram of differentially expressed genes. Differentially expressed genes in blood at 2, 5 and 30 days after WTLI in NHP are shown in the Venn diagram. 25 genes were significantly differentially expressed at all the time points in the study.

We looked for biological processes that were significantly overrepresented among the differentially expressed genes at the various time points using the PANTHER gene ontology program [41, 44]. We found that although more genes were differentially expressed at 30 days (603 genes) than at day 2 (545 genes), there were more biological processes significantly enriched (Bonferroni p-value ≤ 0.05) among the genes at 2 days than those at 30 days, see Table 3. Further comparisons showed that although there were only 81 differentially expressed genes common to days 2 and 30 (Fig 4), all biological processes enriched in changed genes at 30 days were also significantly over represented among those at 2 days (Table 3). Common processes that appeared to be affected throughout the time course were immune system and single organism signaling related to infection. Bacterial response and oxygen containing compounds were significant at 2 days and 30 days after irradiation, but not at 5 days.

**Table 3:** PANTHER Gene ontology analysis of biological processes. Processes that were significantly enriched in differentially regulated genes at a minimum of two time points in the time course.

GO biological process complete	Day 2	Day 5	Day 30
	p-value*	p-value*	p-value*
immune system process	5.33 X10^-31^	1.02 X10^-8^	1.41 X10^-3^
response to stimulus	3.12 X10^-26^	1.52 X10^-5^	1.27 X10^-3^
single organism signaling	2.92 X10^-17^	1.46 X10^-2^	1.74 X10^-4^
defense response	1.99 X10^-23^	5.14 X10^-6^	NS
response to stress	1.82 X10^-21^	4.89 X10^-4^	NS
immune response	1.99 X10^-19^	3.16 X10^-6^	NS
response to molecule of bacterial origin	7.30 X10^-11^	NS	4.45 X10^-2^
response to oxygen-containing compound	1.79 X10^-9^	NS	4.73 X10^-2^

*All p-values are Bonferroni corrected for multiple testing, NS: not significant

The PANTHER gene ontology analysis of the gene expression response in blood cells at the earliest 2-day time point revealed a highly structured and cohesive response to irradiation of the thorax. Biological functions affected at this early time point appeared to reflect a concerted response of the immune system involving activation of almost every blood cell type: platelet, leukocyte, myeloid leukocyte and macrophage activation. Blood coagulation and response to wounding, chemotaxis and leukocyte migration were other processes significant only at 2 days (Table 4) and not at other time points. Child term categories of biological functions such as defense response to Gram-positive bacterium and regulation of tumor-necrosis superfamily production were also observed, suggesting the early activation of specific damage and infection response signaling pathways in blood cells following thoracic irradiation.

**Table 4:** PANTHER biological processes related to the immune response, which are significant at 2 days after WTLI and not significant at later time points.

GO biological process complete	Day 2
	p-value*
cell communication	3.20 X 10^−18^
signal transduction	1.60 X 10^−17^
cell surface receptor signaling pathway	2.57 X 10^−16^
inflammatory response	1.77 X 10^−14^
cell activation	4.42 X 10^−12^
response to bacterium	5.69 X 10^−12^
response to lipopolysaccharide	5.94 X 10^−10^
innate immune response	1.85 X 10^−9^
regulation of tumor necrosis factor superfamily production	2.42 X 10^−9^
blood coagulation	3.78 X 10^−9^
response to wounding	8.12 X 10^−9^
regulation of cytokine production	2.21 X 10^−8^
regulation of body fluid levels	2.22 X 10^−7^
platelet activation	6.35 X 10^−7^
leukocyte migration	7.10 X 10^−7^
regulation of leukocyte activation	8.14 X 10^−7^
platelet degranulation	1.81 X 10^−6^
regulation of programmed cell death	3.81 X 10^−6^
regulation of lymphocyte activation	7.31 X 10^−6^
negative regulation of mononuclear cell proliferation	5.19 X 10^−5^
secretion by cell	8.76 X 10^−5^
leukocyte activation	9.07 X 10^−5^
chemotaxis	1.29 X 10^−4^
defense response to Gram-positive bacterium	2.83 X 10^−4^
myeloid leukocyte activation	5.52 X 10^−4^
endocytosis	6.06 X 10^−4^
cell adhesion	8.61 X 10^−4^
exocytosis	1.13 X 10^−3^
cell migration	1.25 X 10^−3^
macrophage activation	2.10 X 10^−3^

*All p-values are Bonferroni corrected for multiple testing

### Network analysis

Network analysis using IPA revealed a shifting landscape of functional changes across the time course with a few common processes and regulators being involved at all times. We used IPA to predict candidate upstream regulators of the gene expression changes observed and compared their activation/inhibition states at the different post-irradiation times (Fig 5 and S2 Table). We identified 82 candidate regulatory molecules that showed a z score absolute value of at least 2 at a minimum of one time-point in the study. To look at trends in behavior of these transcriptional regulators we also included other time points where the z scores were -2 < z score < 2. This approach allowed us to get an overview of potential changes in gene regulation across the time course, which provide candidate target molecules for future studies, where we may have access to intermediate time point samples and proteins. We classified these 82 regulators into three groups (S2 Table) based on their predicted status at specific times in the study. Group 1 consisted of regulators predicted to be consistently either activated or inhibited at all time-points measured (Fig 5A); Group 2 was defined by a potential change in activity across the time course (Fig 5B); and Group 3 included regulators only predicted to be activated or inhibited at one of the surveyed times (S2 Table).

**Fig 5:** IPA prediction of regulatory molecules. We grouped by these molecule by pattern using the upstream regulator option in IPA and comparing all time-points in the study, which revealed three types of upstream regulators. **A.** Group 1, with persistent activation/inhibition states across the study; **B**. Group 2, regulators that show a trend from activated to inhibited during the course of the study; and Group 3, only activated at one time-point (see S2 Table). All regulators shown pass the z score cut-off absolute value ≥ 2 for at least one time point in the study.

Most of the 21 candidate regulators in Group 1 have known roles in radiation response. In Group 1, which were predicted to be consistently activated/inhibited, TNF (tumor necrosis factor alpha), TGM2 (Transglutaminase 2), IKBKB (inhibitor of kappa light polypeptide gene enhancer in B-cells, kinase beta), HIF1A (hypoxia inducible factor-1A), P38-MAPK (p38 MAP kinase) and cytokines IL5 (Interleukin- 5), IL6 (Interleukin-6) are included, all of which have a known role in radiation or immune response. The microRNA *miR-223*, which is a known regulator of erythroid blood cell development [45], was also predicted as activated with a z score greater than 2 across the time course. The persistently inhibited regulatory factors in Group 1 included DUSP1 (Dual specificity phosphate 1), ER (Estrogen receptor) and Ig (Immunoglobulin) (Fig 5A). Group 2, with 13 members, was the smallest group of candidate regulatory molecules. TGFB1 and TGFB2 (Transforming growth factors beta 1 and 2), IFNG (Interferon gamma), STAT3 (signal transducer and activator of transcription 3,) and PGR (progesterone receptor) are members of this group with IFNG and PGR predicted to be activated at 2 days after WTLI, then inhibited at the intermediate 5 day time-point; and then returning to activation again at 30 days. Group 3 consisted of regulatory molecules only activated/inhibited at one time-point in the time course, suggesting that these specific regulatory molecules may be more time-specific in response to radiation in NHP blood cells. The members of this group are listed in S2 Table.

## Discussion

NHP have been used in radiation dose response studies for many decades [9–11, 17, 46], focusing on the effects of mitigators on acute radiation syndromes of different organ systems and mortality. However, there have been few studies of the cellular and molecular level changes underlying these broad biological end-points. Recently, a few studies have begun to explore the effects of blood cell loss and recovery over time [12] and the transcriptomic response in blood to viral infection [47].

In our study, we used the WTLI model of thoracic irradiation above the midline in NHP, and focused on long-term effects (up to 8 months for micronucleus frequency and up to 30 days for transcriptomics) in blood cells. In a recent retrospective dose-reconstruction study, Prado *et al* [18] calculated that the mean lung and heart dose averaged across 80 NHPs resulting from an average WTLI dose of 10 Gy would be 11.05 Gy and 10.8 Gy, respectively. Since blood flows through the lungs at 2–5 liter minute^-1^ [48], a 10–15 minute lung irradiation protocol will result in uniform irradiation to the blood in *M*. *mulatta* [49]. For our dose and shorter duration of irradiation, we estimate that the dose to the entire blood pool is approximately 10–20% of the dose delivered to the midplane. After the acute dose exposure, irradiated cells would be mixed with newly divided unexposed blood cells over the time course, providing a relevant example of an irradiation scenario that might occur in a radiological event.

Our hematology results show a similar pattern compared to the PBI/BM5 model, where transient decreases in lymphocyte count and platelet count were seen, to a lesser degree than in TBI (11). Our findings with WTLI show a reduced but still-present lymphopenia and thrombocytopenia early on, but differ from the PBI/BM5 model in that a profound neutrophilia is seen approximately 2 months after irradiation, presumably reflecting the response by a largely spared bone marrow pool to radiation-induced pulmonary injury.

To evaluate long-term DNA damage response in the NHP lymphocytes, we used the established human CBMN assay protocol to determine MNi frequency in blood lymphocyte samples collected up to 8 months after initial whole thorax irradiation (Table 1 and Fig 2). Regression analysis showed a significant induction of MNi in the blood lymphocytes across all nine NHPs that persisted with a gradual decline over the 8-month study period, indicating long-term DNA damage in the blood lymphocytes after WTLI (Fig 3). The slow decline in MNi frequency over time may be attributed to the replenishment of mature lymphocytes from damaged and non-damaged progenitor cells in the bone marrow. At 8 months post exposure, we show that MNi frequency remained above baseline. These results are encouraging for the utility of the MNi biomarker in a partial body, long-term animal model. Previously, Gregoire *et al* reported elevated translocation and dicentric chromosome frequencies in blood samples from total body gamma ray irradiated NHPs up to 31 months after irradiation [50] and Thierens *et al* were able to derive dose estimates from dicentrics chromosomes and micronucleus frequencies 6 months after an accidental exposure of a radiological worker [51].

Few studies have used the NHP animal model for cytogenetic biodosimetry. For cytogenetic analyses, the challenge lies in using an optimal culture medium and mitogen where first-division cells are preferred [8]. In the present work, we struggled to score sufficient binucleated (BN) cells in the blood samples collected during the first week post exposure, particularly at 2 days after WTLI (Table 1). These blood samples are likely to include a large proportion of highly damaged mature peripheral blood lymphocytes, which were apoptotic and/or have undergone cell-cycle arrest. The relative MNi yields measured at days 2 and 5 indicate also that the PHA mitogen favored the stimulation of the less damaged lymphocyte cells over the highly damaged cells in the blood cultures. The precipitous drop in lymphocyte numbers by 9 days supports the notion that a large proportion of the circulating lymphocytes had initiated radiation-induced apoptosis and cell death rapidly shortly after WTLI exposure. In the context of a radiological incident or accident where many individuals could receive an acute high-dose partial body exposure of ionizing radiation, future work should look to optimize the CBMN assay culture conditions for increased/improved mitogen-induced cell division of heavily damaged NHP lymphocyte cells.

The blood cells collected from the WTLI irradiated NHPs revealed an overall gene expression response enriched in processes that modulate the immune/inflammatory response to damage and infection, with variations in response at different times. The 2-day response, with 545 genes changing and many biological processes implicated, appeared to be the most dramatic within this time course. At day 2 specifically, processes suggesting blood cell loss, such as negative regulation of mononuclear cell proliferation (p-value = 10^−5^) and platelet activation/degranulation (p-value = 10^−6^) were implicated within both up and down regulated genes. However, at 30 days there were even more responding genes (603 genes, Fig 4), but the biological functions involved at this time were limited to a subset of those at earlier times (Table 3). This suggests that renewal of cells and recovery of normal biological processes and cell numbers may have occurred by 30 days after WTLI. However the immune system remains in a heightened state long after the initial exposure, as suggested by gene expression changes in biological categories related to immune responses (p-values 10^−31^ at 2 days and 10^−4^ at 30 days) and bacterial response (p-values 10^−11^ at 2 days and 10^−2^ at 30 days).

The persistent effect of radiation on transcription in blood cells is seen by examining genes that were significantly differentially expressed at all times in the study. There were 25 such genes, all of which changed in the same direction; either up or down regulated, throughout the study (Fig 6). The up regulated genes contributing to immune response such as *IL1R1* (Interleukin 1 receptor, type 1) (43) and *TLR6* (Toll-like receptor 6) [52, 53], again suggest a persistent alteration of immune response occurring over the course of the 30-day study. This is consistent with previous studies on GI-ARS and H-ARS in NHP where radiation effects were observed on blood cell counts for neutrophils, lymphocytes and platelets, within the first week after TBI [11]; and from PBI/BM5 studies on NHPs in which neutropenia and thrombocytopenia occurred within the first 11 days after irradiation [17]. Further studies on earlier (1 day after irradiation) and intermediate time points such as 7 and 14 days after irradiation, would help to determine if these gene expression and cellular changes fluctuate at intermediate time points, or maintain a steady induction/inhibition level in the 30-day time period as generally appears from the present data.

**Fig 6:** Microarray results of gene expression changes of 25 genes, common across all time points. Gene expression changes of the 25 genes that were differentially expressed at all the time points assayed, the intersection of all groups taken from Fig 4. These genes were selected based on being significantly changed at all times in the study. In each comparison, gene expression signal intensities of these 25 genes at days 2, 5 and 30 were compared with the pre-exposure levels in the matched control to determine fold changes, the bars in the histogram are the mean fold change in five independent biological replicates, error bars are SEM. The dashed line represents the normalized pre-exposure expression level.

We validated changes in levels of mRNA for two up and two down regulated genes as measured by microarrays (Fig 6), using real-time qRT-PCR (Fig 7). The genes we measured were *IL1R* and *LY96* (Lymphocyte antigen 96/Myeloid differentiation factor 2), which were consistently up regulated after irradiation; and *MARCKSL1* (Myristoylated alanine-rich C kinase substrate-like 1) and *FAIM3* (Fc fragment of IgM receptor), which were down regulated after irradiation. We found that measurements using PCR closely correlated with microarray fold changes for most time points and genes measured.

**Fig 7:** qRT-PCR validation of gene expression changes. Gene expression was measured in blood cell RNA using qRT-PCR to validate the microarray measurements. Two consistently up regulated genes are shown here, *IL1R1* (A) and *LY96* (B); and two downregulated genes, *MARCKSL1* (C) and *FAIM3* (D). Relative expression are mean fold changes at 2, 5 and 30 days in at least three biological replicates. Microarray changes are solid symbols (●) and qRT-PCR fold changes are shown in open symbols (o), representing the mean, error bars are SEM.

Using a network approach, we identified several strong candidate regulators of the transcriptional changes observed over the 30-day time course (Fig 5). Information of networks and signaling pathways based on gene expression changes could facilitate the understanding of the nature of the biological response to radiation and the changes over time. We grouped the potential regulators into three categories based on patterns of response. Group 1 included predicted upstream regulators with consistent activation/inhibition states at all the time points in this study. This group includes transcriptional regulators such as transglutaminase 2 (TGM2), an enzyme that leads to activation of transcription factors NFκB and HIF1β through a transamidation reaction [54], and which is involved in cell fate of blood cells [55, 56]. This is a novel regulator in ionizing radiation response in blood cells. Also in Group 1 were well-known radiation response regulators such as TNF proteins, interleukins (IL1B, IL5 and IL6) and hypoxia response regulator HIF1A [57–59]. IKBKB (which is a negative regulator of NFkB) and p38MAPK; were also predicted to be activated and may have a role in the radiation response in blood cells [60, 61]. CSF2, also called GM-CSF (granulocyte-macrophage colony stimulating factor) was in Group 1, as a predicted persistent activator of genes. CSF2 is well known for its ability to counter myelosuppression [62] and is administered after radiological events to boost and activate the immune response to infection [63]. Our results indicate that endogenous CSF2 activation may occur after partial body irradiation. The microRNA *miR-223*, known to be involved in red blood cell development via LMO2 (LIM-only protein 2, rhombotin-like 2) [45] was predicted to lead to both up and down regulation of specific transcripts in the study. Surprisingly, in our study most potential downstream targets of *miR-223* were up regulated at the mRNA level rather than the expected repression of genes by microRNA mediated silencing. It is possible that current information about the indirect targets of microRNA *miR-223* is incomplete and that an intermediate transcriptional regulator may be responsible for its potential role as a transcriptional activator [64, 65].

We also observed another interesting pattern in the prediction of transcriptional regulators, where the state of the regulator might switch from activated to inhibited, and then back again, over the time course. Most striking were the predicted responses of IFNG (Interferon G) and PGR (progesterone receptor), which changed from activated to inhibited and then activated again at 2, 5 and 30 days after irradiation, respectively (Fig 5B). We also looked for other known regulators involved in oxidative stress after radiation and NRF2 (NFE2L2, Nuclear Factor, erythroid 2 like 2) which is a transcription factor that induces gene expression of protective genes against oxidative stress, and was predicted to be activated at 2 days after irradiation. This is a central player in cellular defense against xenobiotics and oxidative damage [66] and the early activation of this transcription factor may indicate high levels of oxidative damage in the initial response to radiation. Further studies on intermediate time points and complementary cellular/physiological results could clarify the role of these types of regulators and their role in the radiation response in blood.

Taken together, our study is an important first step in our understanding of the long-term cellular and molecular response to partial body irradiation using the NHP WTLI model. The MNi biomarker showed a robust response to high-dose partial body irradiation and has potential for cytogenetic biodosimetry studies to estimate absorbed dose weeks after a radiological incident or accident. Future studies should look to validate this biomarker for long-term retrospective dose estimations. The gene expression response in blood cells up to a month after partial body irradiation revealed a combination of persistent and time-point specific changes indicating that the earliest change (measured in this study) is also the strongest response. The gene expression changes suggested enrichment of processes related to blood cell loss at 2 days after exposure. Following this, at 5 days after irradiation, the immune response was persistent and included specific genes that suggest mechanisms responding to infection and single organism signaling remain affected. At 30 days after irradiation, changes in immune response genes appear to be maintained; however, blood cell counts show that non-immune, neutrophil-mediated responses to tissue injury and possibly bacterial infection predominate, waning as pulmonary injury progresses from pneumonitis to fibrosis. Further studies are required to elucidate how the biological response evolves over time. The long-term effects of radiation at the transcriptomic level corroborate the observed physiological changes in blood cells, and could be useful in identifying potential drug targets for future mitigator studies.

## Supporting information

S1 Table Significantly differentially regulated genes. Gene lists of differentially expressed genes at all time-points in the study.
(XLSX)

S2 Table IPA regulatory factor analysis. Complete list of IPA generated upstream regulators with z-scores, based on network analysis of gene lists and expression changes at days 2, 5 and 30.
(XLSX)
